RETRACTED

# Injuries in College Basketball Sports Based on Machine Learning from the Perspective of the Integration of Sports and Medicine

**DOI:** 10.1155/2022/1429042

**Published:** 2022-06-14

**Authors:** Dongming Zhao

**Affiliations:** Department of Physical Education, Guizhou University of Finance and Economics, Guiyang 550025, Guizhou, China

## Abstract

Basketball is one of the popular sports in colleges. Basketball injuries are a common thing, and the use of machine learning and other technologies can effectively reduce basketball injuries, which should start with prevention. Nonstandard basketball movements and lack of physical coordination will not only reduce sports efficiency for athletes but also increase the probability of injury. Therefore, effective reduction and targeted prevention of nonstandard actions are of great significance to college basketball. With the development of science and technology, artificial intelligence technology is closer to our lives. Based on the machine learning platform, this paper studies basketball injuries from the perspective of the integration of sports and medicine. Research on what aspects cause college students' basketball injuries is needed for the future. Effectively preventing college students from being injured in basketball is an urgent problem in the field of sports medicine. To find the most suitable machine learning platform for college basketball injury research, this article will introduce three different methods for comparative analysis. The techniques used in the experiment in this paper are traditional BP neural network technology, SCG neural network technology, and RBF neural network technology. Through experiments, it is known that, through experiments, RBF neural network technical prediction accuracy rate is as high as 95.4%, which is a relatively good neural network algorithm for studying the basketball loss of college students.

## 1. Introduction

Basketball injuries, as the name suggests, are injuries that occur while playing basketball and are widespread in the sports world. Basketball injuries are closely related to sports training, sports technology, sports items, sports training level, and sports environment. As colleges and universities pay increasingly attention to the athletic ability of college students, the competitive level of college basketball games is also getting higher and higher, and the intensity of confrontation is becoming increasingly intense. With the increasing training pressure, the probability of injury to college basketball players is also increasing. Due to the high intensity of basketball sports, injuries in sports affect the future development of college students to a large extent. The impact of basketball injury can be terrifying. An unfortunate injury to an athlete can have unimaginable consequences for the individual, their team, and their family. Sports injuries will not only make athletes unable to participate in high-intensity training and competitions, but also cause athletes to be disabled or even be life-threatening in severe cases. At the same time, it brings a certain psychological burden to athletes and hinders the development of their sports. Therefore, the field of basketball sports injuries is worthy of our in-depth study to avoid. Basketball injuries focus on prevention. There are many reasons for sports injuries although prevention is always emphasized, but sometimes athletes play too frequently, and basketball sports injuries are difficult to avoid. Therefore, it is essential to guide college students to prevent sports injuries in basketball. This is of great significance to promoting the development of basketball and protecting the health of basketball players.

RETRACTED

This paper focuses on college basketball injuries and is based on machine learning theory. Compared with the ordinary research on college basketball injury, this paper has the following innovations: (1) it proposes a machine learning method. The general way to study college basketball injuries is through expert interviews and mathematical statistics. It always stays at the level of interviewing and researching through people. Based on machine learning, this paper makes basketball injury research systematic and sustainable and greatly reduces the cost of personnel interviews. (2) This paper uses a variety of neural network techniques to study the injury of college basketball. Through systematic research of multimethods, the advantages and disadvantages of each method are compared, and a neural network method most suitable for college students' basketball injury is found. This makes the research results more reliable and authoritative. Therefore, this study is innovative.

## 2. Related Work

With the development and continuous improvement of artificial network technology, increasing people have studied the research of college basketball injury based on machine learning. Among them, Shimoura et al.'s study aimed to investigate the relationship between FMS scores and injury in basketball players, and the participants were 81 male college basketball players (mean age, 20.1 ± 1.3 years). According to the research and development results, it can be concluded that the FMS score of basketball players decreases with the increase of injuries [1]. Wehsener research was to develop a unique repair method for the fracture problem of college female basketball players [2]. Helma et al. proposed through experiments that the use of deep learning knowledge can solve the problem of blurred visual appearance in 2.5D games [3]. Li and Zhang improved the shooting accuracy in basketball through an improved line radial basis function neural network [4]. Alderden et al. established a model of pressure injury development through experimental studies, dividing the recorded data into training (67%) and test (33%) datasets. It also uses the random forest algorithm through the R package to develop models to predict the risk of pressure injury [5]. Wang studied the structure of the exercise brain machine and improved it on the basis of traditional methods. Furthermore, powered by machine learning and SVM techniques, it uses DSP filters to convert the preprocessed EEG signals *X* into time series [6]. Wang and Gao used machine learning technology to build a basketball motion feature recognition model [7]. Thabtah et al. proposed a new intelligent machine learning framework through research, selecting several machine learning methods that utilize different learning schemes to derive models. It includes Naive Bayes, Artificial Neural Networks, and Decision Trees for predicting the outcome of basketball games. It aims to discover influential feature sets that influence basketball game outcomes [8].

RETRACTED

Inspired by other researchers, it identified pain points in college basketball and completed a machine learning-based conceptual design. It identifies some actions in basketball that are likely to cause injury to players and the associated algorithms for calculating basketball injuries. The validity of its function and the rationality of its design are verified by developing a machine learning-based basketball injury research experiment for college students from the perspective of CIN-Physical Medicine Integration. Its deficiency lies in the use of neural network technology to deduce the cause of basketball injury through the objective data import system. Its scientific demonstration method can be used for reference in this research. However, there are still shortcomings in judging the cause of basketball injuries only through data reflection. After all, neural network technology also has errors and cannot completely replace the experience guidance of the coaching staff.

## 3. Machine Learning-Based Basketball Injury Prevention Method

### 3.1. Neural Networks

#### 3.1.1. Definition and Characteristics of Artificial Neural Network

Artificial Neural Network (ANN) is referred to as Neural Network (NN). It is based on a biological neural network, a mathematical model imitating the response mechanism of the human brain to external stimuli [9]. The model is characterized by the ability to handle concurrency, high fault tolerance, intelligence, and self-learning. It combines information processing and storage and has attracted the attention of many disciplines through its unique adaptive learning capability. In principle, it is a system of many node structures. The complex network formed has nonlinear characteristics, which can deal with complex logic operations and systems realized by nonlinear relationships and can effectively deal with the problem of basketball injuries. It reflects the function of the human brain; however, it is not the real human brain, but an abstraction of the function of the human brain.

RETRACTED

#### 3.1.2. Artificial Neuron Model

A neural network is a mathematical plus Internet model. Its internal structure is a large number of nodes connected to each other. The schematic diagram of the neuron is shown in Figure 1. Each node represents an output function called an activation function [10]. Each connection between two nodes has a weighted value, called weight [11]. In this way, the neural network simulates the scene of the human brain recalling things. The output of the network largely depends on how the network is connected, its structure, weights, and activation functions. Neuron processing units can represent different objects. Generally, processing units can be divided into three categories: input units, output units, and hidden units [12]. The input unit is to receive signals and data from the external space. The output unit is used to realize the result of output system processing. Hidden units exist between the input and output units. The weights represent the connection strength between hidden units. Artificial neural networks can be understood as a kind of adaptability, imitating the information processing method of the brain and simulating the ability of the human brain nervous system to process complex information, which can solve the problem of basketball injuries very well.

Neurons have nonlinear input and output capabilities, as well as plasticity. Neuron weights can be adjusted and are generally multi-input and unilateral output models. According to this characteristic, the artificial neuron model can be constructed as shown in Figure 2. Among them, *w* is the connection weight between several other neurons and the *i*th neuron in the previous layer, *θ* is the threshold of this neuron, and *u*_1_ is the neuron's processing process.

A neuron consists of three parts: input, processing, and output. It receives the signal input from the outside of the system or the signal output by other neurons as its own input content and then outputs the processing result in the form of a signal to other neurons or outside of the system. The relationship of each variable is

(1) $$\begin{array}{c} \nu_{a}=\sum_{j}w_{ab}x_{b}+h_{a}, \end{array}$$

(2) $$\begin{array}{c} y_{a}=f\left(v_{a}\right). \end{array}$$

Among them, *w*_*ab*_ is the connection weight of the input terminal, that is, the binding strength, and *y*_a_ is the output signal. *h*_a_ is the closed value, *v*_*a*_ represents the internal state of the neuron, *x*_b_ is the input signal, and *f* is the activation function, and *j* represents the number of neurons.

RETRACTED

#### 3.1.3. Basic Structure of Neural Network

The complexity of the basic structural connections of neural networks corresponds to the diversity of their types. This article presents several representative structures. According to the network topology, it is divided into layered network and mesh network. According to the characteristics of information transmission, it can be divided into feedforward network and feedback network. The following is an introduction to these types of networks:

*(1) Layered Networks and Mesh Networks*. The layered network model is connected in the order of layers. Each layer is only related to the adjacent layers, and the neurons of each layer are connected to the neurons of the upper and lower layers. This is conducive to the transmission of information within the network [13]. Each neuron in the mesh network model structure is connected to any neuron in the network. This structure allows information to propagate to each neuron, as shown in Figure 3.

*(2) Feedforward Network and Feedback Network*. The next-level neurons in the feedforward network must receive the input of the previous layer of neurons. There is no feedback behavior in this network structure. Each neuron in the network has an output direction that is downward. The main feature of this network structure is simple and easy to implement [14]. In a feedback network, each unit is a multiple-input single-output model. The specific structure is shown in Figures 4 and 5.

#### 3.1.4. Learning of Neural Network

Neural networks are complex interconnected systems of networks. The complex connections of neurons lead to the way information is transmitted in the network. Therefore, generally, after the network structure is determined, the connection weights need to be adjusted. It is done by using training. Network learning algorithms are the core part of neural network intelligence. Learning methods are divided into tutored learning and tutorless learning.

*(1) There Is a Tutor to Learn*. The learning method is provided by the tutor with training data. The tutor compares the error between the expected output and the actual output of the network. It modifies the weights of each connection according to the error and then finds the appropriate connection between the input and the output through the adjustment of the weights. When the input random samples are infinitely guided by the tutor, the actual output of the network model can approach the output expectation [15].

*(2) Learning without a Tutor*. Learning without a tutor has no target output, only training data through input, and the learning process is a self-organizing process, learning and improving the network system by continuously inputting data [16].

RETRACTED

BP neural network is a way of tutoring learning. Taking a typical three-layer BP network as an example, the general process of neuron learning is shown in Figure 6. The initial neural network weights are generally random numbers. The learning of the network is achieved by adjusting the weights of neurons. The learning process consists of two processes of signal transfer from top to bottom and error transfer from bottom to top [17]. Forward propagation is that the input samples enter from the input layer, specify the weights of neuron nodes, and carry out forward propagation from the hidden layer to the activation function and then to the output layer. If the expected output is far from the actual output, the network switches to a backpropagation mode of error. To introduce the error into the hidden layer and propagate to the input layer, the internal action continuously modifies the weight of each neuron node [18]. The forward propagation of the error and the backward propagation of the error are not carried out independently in the BP algorithm's learning phase but are completed in a loop at the same time. The BP network's training and learning process is the process of regularly modifying the weights. The learning process is repeated until the actual output falls within an acceptable range of the desired output.

### 3.2. BP Neural Network Algorithm

Error backpropagation learning algorithm (referred to as BP algorithm) is a multilayer feedforward neural network algorithm for corrective learning. It has a wide range of applications and is a relatively mature network model. Since the BP network was proposed in 1986, the theory and methods have been continuously improved during the period. Therefore, the BP network has been developed rapidly. BP network is an error propagation algorithm of some sort. The input layer, hidden layer, and output layer are the three layers that make up the topology structure of the BP neural network model.  Figure 7 is a typical three-layer forward network structure.

Among them, *X* is the input layer vector, and *O* is the output layer vector. Input vector *X*=(*x*_1_, *x*_2_,…,*x*_*n*_)^*T*^, where *X*_0_ = −1 is the threshold set for the hidden layer neurons. The output vector *Y*=(*y*_1_, *y*_2_,…,*y*_*m*_)^*T*^ of the hidden layer, where *Y*_0_ = −1 is the threshold setting for the output layer neurons. The output vector *O*=(*o*_1_, *o*_2_,…,*o*_*n*_)^*T*^ of the output layer, and the expected output vector *r*=(*r*_1_, *r*_2_,…,*r*_*n*_)^*T*^. The weight matrix *T*=(*t*_1_, *t*_2_,…,*t*_*m*_)^*T*^ from the input layer to the hidden layer, and the column vector *T*_j_ is the weight vector corresponding to the *j*th neuron in the hidden layer. The weight matrix *Z*=(*z*_1_, *z*_2_,…,*z*_*k*_)^*T*^ implied to the output layer, and the column vector *Z*_k_ is the weight vector corresponding to the kth neuron in the output layer.

RETRACTED

For the output layer, there is the following formula, where *k*=1,2,…, *n*:

(3) $$\begin{array}{c} o_{k}=f\left({\text{net}}_{k}\right)=f\left(\sum_{j=0}^{m}z_{jk}y_{j}\right). \end{array}$$

For the hidden layer, there is the following formula, where *j*=1,2,…, *m*:

(4) $$\begin{array}{c} y_{j}=f\left({\text{net}}_{j}\right)=f\left(\sum_{i=0}^{n}t_{ij}x_{i}\right). \end{array}$$

In formulas (2) and (3), the net represents a neural network.

The *f* function of the above formula is a unipolar function:

(5) $$\begin{array}{c} f\left(x\right)=\frac{1}{1+e^{-x}} \end{array}$$

Since *f*(*x*) is continuously differentiable,

(6) $$\begin{array}{c} f^{\prime }\left(x\right)=f\left(x\right)\left[1-f\left(x\right)\right]. \end{array}$$

When the actual output is not equal to the expected output, there is an error *E*. The formula is as follows:

(7) $$\begin{array}{c} E=\frac{1}{2}{\left(r-O\right)}^{2}=\frac{1}{2}\sum_{k=1}^{2}{\left(r_{k}-O_{k}\right)}^{2}=\frac{1}{2}\sum_{k=1}^{1}{\left(r_{k}-f\left(\sum_{j=0}^{m}z_{jk}y_{j}\right)\right)}^{2}. \end{array}$$

(8) $$\begin{array}{c} E=\frac{1}{2}{\sum_{k=1}^{1}\left\{r_{k}-f\left[\sum_{j=0}^{m}z_{jk}f\left(\sum_{i=0}^{n}t_{ij}x_{i}\right)\right]\right\}}^{2}. \end{array}$$

According to the formula of the error *E*, the error is a function of the weights *w*_*jk*_ and *v*_*ij*_ of each layer. Therefore, adjusting the weights can change the error *E*. The weights are generally adjusted with small aspects, namely,

(9) $$\begin{array}{c} \Delta_{jk}=-\eta \frac{\partial E}{\partial z_{jk}}=-\eta \frac{\partial E}{\partial n\;et_{k}}\frac{\partial n\;et_{k}}{\partial z_{jk}}. \end{array}$$

(10) $$\begin{array}{c} \Delta t_{ij}=-\eta \frac{\partial E}{\partial t_{ij}}=-\eta \frac{\partial E}{\partial n\;et_{j}}\frac{\partial n\;et_{j}}{\partial t_{ij}}. \end{array}$$

Among them, *j*=1,2,…, *m*, *k*=1,2,…, *n*, *i*=1,2,…, *n*, *η* represents the error factor.

RETRACTED

The error signal is defined separately for the output layer and the hidden layer. The formula is as follows:

(11) $$\begin{array}{c} \delta_{k}^{o}=-\frac{\partial E}{\partial n\;et_{k}}=-\frac{\partial E}{\partial o_{k}}\frac{\partial o_{k}}{\partial n\;et_{k}}=-\frac{\partial E}{\partial o_{k}}f^{\prime }\left(net_{k}\right), \end{array}$$

(12) $$\begin{array}{c} \delta_{j}^{y}=-\frac{\partial E}{\partial n\;et_{j}}=-\frac{\partial E}{\partial y_{j}}\frac{\partial y_{j}}{\partial n\;et_{j}}=-\frac{\partial E}{\partial y_{j}}f^{\prime }\left(net_{j}\right). \end{array}$$

It computes the partial derivative of the network error with respect to the output of each layer. The output layer and hidden layer are as follows:

(13) $$\begin{array}{c} \frac{\partial E}{\partial y_{j}}=-\sum_{k=1}^{n}\left(r_{k}-o_{k}\right)f^{\prime }\left(net_{k}\right)z_{jk}. \end{array}$$

(14) $$\begin{array}{c} \frac{\partial E}{\partial o_{k}}=-\left(r_{k}-o_{k}\right). \end{array}$$

It substitutes formulas (13) and (14) into formulas (11) and (12) to get

(15) $$\begin{array}{c} \delta_{k}^{o}=\left(r_{k}-o_{k}\right)o_{k}\left(1-o_{k}\right), \end{array}$$

(16) $$\begin{array}{c} \delta_{j}^{y}=\left[\sum_{k=1}^{n}\left(r_{k}-o_{k}\right)f^{\prime }\left(net\right)z_{jk}\right]f^{\prime }\left(net\right)=\left(\sum_{k=1}^{n}\delta_{k}^{o}z_{jk}\right)y_{j}\left(1-y_{j}\right). \end{array}$$

Combining the above formulas (15) and (16) with formulas (4), (11), and (12), it can be concluded that the weight adjustment formula of the BP learning algorithm is

(17) $$\begin{array}{c} \Delta z_{jk}=\eta \delta_{k}^{o}y_{j}=\eta \left(r_{k}-o_{k}\right)o_{k}\left(1-o_{k}\right)y_{j}. \end{array}$$

(18) $$\begin{array}{c} \Delta t_{ij}=\eta \delta_{j}^{y}x_{i}=\eta \left(\sum_{k=1}^{n}\delta_{n}^{o}z_{jk}\right)y_{j}\left(1-y_{j}\right)x_{i}. \end{array}$$

In summary, the BP algorithm is roughly described as follows: it initializes the network and determines the weights and assigns a random number to the node weights and neuron thresholds of the hidden layer and output layer. And it feeds its input and desired output into the network through training. By calculating the output error *E* of the network, it checks whether *E* meets the accuracy requirements. If the exact value is reached, end the study; otherwise, continue to repeat the study steps until the desired output is reached, and end the study.

### 3.3. Quantized Conjugate Gradient Neural Network Algorithm (SCG Neural Network)

In the 1950s, scientists proposed the conjugate gradient method. After more than ten years of development and improvement, the experimenters proposed the conjugate gradient method for nonlinear optimization problems on this basis. Now, it has been widely developed in various fields. Conjugate gradient method is an improved method based on BP neural network. It has the advantages of fast convergence and quadratic termination. Each search direction is conjugated to each other. Therefore, the storage capacity of this algorithm is small, and the calculation is convenient. The conjugate gradient neural network algorithm selects the second-order Taylor expansion of the function as the function approximation, and the BP algorithm selects the first-order Taylor formula as the function approximation, so the conjugate gradient algorithm is compared to the BP algorithm. It is orders of magnitude faster and can handle complex basketball injury data.

RETRACTED

The algorithm principle is as follows: it sets the quadratic function as *f*(*x*)=*H*+*d*^*T*^*X*+1/2*X*^*T*^*GX*, where H is a constant, *d* and *X* are *n*-dimensional column vectors, *G* is a symmetric positive definite matrix, the conjugate gradient method is used to find the minimum point of the function *f*(*x*), and *T* represents the transposition.

The first step in the exploration of the conjugate gradient method is to find *X*(*a*+1) in the direction of *S*(*a*)=−∇*f*(*X*(*a*)) along the negative gradient direction *X*(*a*), and let *S*(*a*+1)=−∇*f*(*X*(*a*+1))+*β*^*a*^*S*^*a*^.

The above formula *β*^*a*^ makes two non-zero vectors *S*^*a*^ and *S*^(*a*+1)^ in the *n*-dimensional Euclidean space conjugate with respect to the *A* matrix, namely,

(19) $$\begin{array}{c} {\left[S\left(a+1\right)\right]}^{T}AS^{a}=0. \end{array}$$

Among them, *a*=0,1,2,…, *n* − 1.

Since ∇*f*(*x*)=*d*+*GX*, let

(20) $$\begin{array}{c} g\left(a\right)=\nabla f\left(X\left(a\right)\right)=d+GX\left(a\right), \end{array}$$

(21) $$\begin{array}{c} g\left(a+1\right)=\nabla f\left(X\left(a+1\right)\right)=d+GX\left(a+1\right). \end{array}$$

Subtracting the two formulas, it can get

(22) $$\begin{array}{c} g\left(a+1\right)-g\left(a\right)=G\left(X\left(a+1\right)-X\left(a\right)\right). \end{array}$$

In *a* + 1 iteration, there are

(23) $$\begin{array}{c} X\left(a+1\right)=X\left(a\right)+\alpha \left(a\right)S\left(a\right). \end{array}$$

Substituting this into formula (23), it can get

(24) $$\begin{array}{c} g\left(a+1\right)-g\left(a\right)=G\alpha \left(a\right)S\left(a\right). \end{array}$$

Among them, *a*=0,1,2,…, *n* − 1, exp is an exponential function with the base of a natural constant *e*.

In the formula, *α*(*a*) is the optimal step size of +1 iteration.

### 3.4. Radial Basis Function Neural Network Algorithm (RBF Neural Network)

RBF is a mathematical mode of difference processing of functions in a multidimensional space. The RBF neural network belongs to the multilayer feedforward neural network model, and Figure 8 is its network structure diagram. The activation function of the neuron is a nonlinear local response function that is symmetrical to the center. The sigmoid function used by the BP network is a global response function. The radial basis function is used by the RBF network. The direction basis function affects the results only when the input falls within a specific range of the input space, which greatly reduces the time complexity of the RBF network, which is very suitable for basketball injury research. Therefore, the RBF network is 3–5 orders of magnitude faster than the ordinary BP network.

RETRACTED

The performance of an RBF neural network depends on the learning algorithm used. The learning algorithm needs to determine three important parameters. These include the central function, variance, and weights. The method has two stages, including using an unsupervised learning algorithm to determine the center and response radius of the radial basis function and using a mentored algorithm to determine the weights.

The mathematical model used by the radial basis function in the RBF neural network is a Gaussian function. Therefore, the activation function of the hidden layer neurons of the RBF neural network is expressed as

(25) $$\begin{array}{c} \varphi \left(a_{r}-b_{i}\right)=\exp\left(-\frac{1}{2\sigma^{2}}{\left\|a_{r}-b_{i}\right\|}^{2}\right). \end{array}$$

Among them, *a*_*r*_ represents the *r*th input data, *b*_*i*_ represents the *i*th center vector, ‖*a*_*r*_ − *b*_*i*_‖ represents the Euclidean norm, and exp is an exponential function with the base of natural constant *e*.

Then, the output representation formula of the RBF neural network is as follows:

(26) $$\begin{array}{c} y_{i}=\sum_{i=1}^{k}w_{ij}\exp\left(-\frac{1}{2\sigma^{2}}{\left\|a_{r}-b_{i}\right\|}^{2}\right). \end{array}$$

Among them, *j*=1,2,…, *N*. The weight from the *i*th node of the hidden layer to the *j*th node of the output layer is denoted by *w*_*ij*_. The number of nodes in the hidden layer is denoted by *k*. The output of the *j*th node of the output layer is denoted by *y*_i_. The total number of samples is *N*.

## 4. Experiment of College Basketball Injury Based on Machine Learning

This experiment is completed on the data mining platform by calling the MATLAB algorithm interface for secondary development. The experiments used in this system are all completed through simulation experiments.

Introduction to MATLAB: MATLAB means matrix factory. The software is a high-tech computing environment for scientific computing, visualization, and interactive programming. It provides scientific and effective calculations for scientific research through data simulation technology. It provides a reliable problem-solving model in numerous domains.

RETRACTED

Through the way of questionnaires, the injured parts of college basketball players are obtained as shown in Table 1. Sports injuries in college basketball are extensive. Among them, the injured parts of different college players' basketball positions are also roughly different.

According to Table 1, the total number of 211 cases of college basketball players' defender injuries was obtained. Among them, the knee is the most serious injury, accounting for 21.3% of the total number of defenders injured. Next is the ankle joint, with 28 injuries, accounting for 13.3% of the guard's total injuries. Calf injuries ranked third, with 25 injuries accounting for 11.8% of the guard's total injuries. The wrist and forearm injuries were both 16, accounting for 7.6% of the guard's total injuries.

Similarly, the total number of striker injuries of college basketball players is 220 cases. Among them, the knee joint was the most serious, with 58 injuries, accounting for 26.4% of the striker's total injuries. Next is the ankle joint, with 51 injuries, accounting for 23.2% of the striker's total injuries. Calf injuries ranked third with 29, accounting for 13.2% of strikers' total injuries. Back and spine injuries ranked fourth with 19, accounting for 8.7% of all forward injuries. Last is the foot, with 16 injuries, accounting for 7.3% of strikers' total injuries.

In the same way, the total number of center injuries of college basketball players is 153 cases. Compared with defenders, forwards have slightly fewer players but have the most ankle injuries, with 40 injuries, accounting for 26.1% of the total injuries for centers. Followed by the number of knee injuries, the number of injuries was 36, accounting for 23.5% of the total number of injuries to the front center. The number of calf injuries ranked third, with 16 injuries, accounting for 10.5% of the total injuries at the center. Back and spine injuries were the fewest at 11, accounting for 7.2 percent of all injuries in centers.

### 4.1. Simulation Samples

The sample data are all from real college students. This is for the optionality of the test to select samples without subjective factors. And the sample cannot be too biased; for example, it can not select all athletes who will be the samples of this experiment. All in all, it is about making the sample random and fair.

#### 4.1.1. Acquisition of Simulation Samples

In the machine learning model system, it is necessary to select experimentally meaningful data without artificial interference with the experiment. The sample used in this study is based on raw data from 300 college basketball players for evaluation. The system uses a five-level system: health, minor injuries, moderate injury, advanced injuries, and serious injuries. The rules for the system to process samples are as follows. The indicators are converted into 5, 4, 3, 2, and 1, respectively, for healthy, minor injury, medium injury, advanced injury, and serious injury. The output health, minor injury, medium injury, advanced injury, and serious injury correspond to 5 intervals, namely, [4.5 5], [4 4.5], [3.5 4], [3 3.5], [0 3].

RETRACTED

In the experiment, the data of 300 samples were compared and analyzed. The valid sample set is taken from 275 student data. It divides these valid sample data into a test sample set and training sample set. The training samples of this experiment are taken from random data of 240 college students. The test sample set is taken from the remaining student data and used to test and train the resulting neural network model.

#### 4.1.2. Correlation of Simulation Samples

In the college basketball injury system based on machine learning, there must be some indicators that affect the system results. And some indicators even have a negligible impact. Faced with negligible indicators during the experiment, they can be appropriately discarded during data input to achieve the purpose of dimensionality reduction. The purpose of correlation analysis is to make the main feature clear when the main eigenvalue is ambiguous. In this way, the main feature information is also easily recognized by the system, which can effectively improve the system recognition rate. In addition, due to the reduction of the dimension of the input vector, the number of nodes in the network structure will be correspondingly reduced, and the complexity of the network will be reduced. This is a good solution to the trouble caused by too many network dimensions.

According to the relevant researches, the nearest neighbor algorithm can determine the relevant properties. Therefore, the nearest neighbor algorithm was used in this experiment to judge the relationship between injuries in college basketball sports in the event of pinching, heavy weight, intense confrontation, excessive use of lower limbs, body collision in the air, nonstop acceleration, emergency stop jump shot, number of blocked shots, loss of center of gravity, fast dribbling speed, excessive exercise time, insufficient rest, ill-fitting shoes, alcohol and smoking, and other indicators. The following data were obtained through systematic analysis, and the details are shown in Table 2.

RETRACTED

From Table 2, intuitively, the degree of correlation between each index and college basketball injury can be seen. Each index has a significant impact on the results of the system evaluation. And the output dimension of this system is not high. Therefore, the experiment will select all above indicators as the input of the college basketball sports injury research for modeling.

#### 4.1.3. Validity Analysis of Simulation Samples

Due to the need to ensure the validity of the sample data used to build the model, this experiment uses cross-validation to select experimental sample data, especially when the total number of samples is not large enough.

This experiment adopts the principle of *k*-fold cross-validation: divide the data into *k* equal parts. Each time the experiment is run, one of these will be selected as the test set. The rest of the samples are all used as the training set, and the process is repeated *k* times, so that each test data is tested exactly once. The correct rate of the experiment is averaged over the sum of *k* validations.

Since the number of samples is not large, this experiment adopts 5-fold cross-validation, that is; the 275 groups of sample data are randomly divided into 5 equal parts. A total of 55 sets of data are used as the test set, and the remaining 220 sets of data are used as the training set. It is also used for 5-fold cross-validation for BP neural network and SCG neural network and RBF neural network, respectively. The result is as follows:

The results based on the BP neural network model are shown in Table 3.

The data simulation is carried out on the basketball injury model of college students based on SCG neural network. It uploads the simulation sample data to the test system for experiment and obtains the following data. Details are shown in Figure 9.

Through the experimental test, it can be concluded that the data accuracy rate of college basketball injury model based on SCG neural network is 91.4%, which has reached a high level.

The data simulation of college basketball injury model based on RBF neural network is carried out. It uploads the simulation sample data to the test system for experiment and obtains the following data. The details are shown in Figure 10.

From the experimental data in Table 3 and Figures 9 and 10, the average correct positive rates of 5-fold cross-validation based on BP neural network, SCG neural network, and RBF neural network are 78.2%, 83.3%, and 85.1%, respectively. The accuracy rate is relatively high. This proves that the filtered sample data can meet the modeling requirements of this experiment. Through the experimental comparison, it can be concluded that the data accuracy rate of college basketball injury model based on RBF neural network is 95.4%, which has reached a very high level.

RETRACTED

### 4.2. Comparison of Test Results

By comparing the accuracy of cross-checking and model testing based on BP neural network, SCG neural network, and RBF neural network, Figure 11 shows the comparison results. It can be seen that the recognition effect based on the RBF neural network is the best.

## 5. Discussion

As colleges and universities pay increasingly attention to the development of sports, the risk of college students' injury in sports also increases. It uses artificial neural network knowledge and research on college basketball injuries to predict the risk of college basketball injuries. The experiments are carried out through modeling and analysis of several different neural network algorithms. It is tested by importing real data, and the advantages and disadvantages of several different algorithms are compared and analyzed. Thus, a neural network model most suitable for college basketball injury is obtained. In the era of intelligence, artificial neural network technology is used in all aspects of our lives. Using neural network technology as a medium, combining sports and medical fields can scientifically reduce sports injuries to a minimum.

## 6. Conclusions

Through experimental research, the following conclusions are drawn: (1) using neural network technology and inputting the indicator data of college basketball players, the system can predict college basketball injuries after continuous learning. Through cross-checking, we know that the cross-validation rate of the neural network technology used in this paper is more than 70%, which can well predict college basketball injuries. (2) By comparing the BP neural network, the SCG neural network, and the RBF neural network, the most accurate prediction accuracy rate is the system based on the RBF neural network. The expected output is very close to the predicted output, and its accuracy is as high as 95.4%. However, this study still has shortcomings; that is, the prediction accuracy cannot be infinitely approached at 100%, which means that when the input data is too large, there will be a lot of inaccurate data prediction, which need to be improved. In addition, this experiment only uses three neural network methods for testing experiments. There are not enough methods, and there may be better neural network methods to achieve higher prediction accuracy. Therefore, improving the prediction accuracy of the system is the direction of future research.

## Figures and Tables

**Figure 1:** Schematic diagram of a neuron.

RETRACTED

**Figure 2:** Artificial neuron model diagram.

**Figure 3:** Layered structure and network structure diagram: (a) Layered network; (b) mesh network.

**Figure 4:** Feedforward network structure diagram.

**Figure 5:** Feedback network structure diagram.

**Figure 6:** Diagram of neural network learning process.

**Figure 7:** Three-layer forward network structure diagram.

**Figure 8:** Three-layer forward network structure diagram.

**Figure 9:** Data test chart of college basketball injury model based on SCG neural network. (a) SCG neural network college basketball injury data map. (b) SCG neural network average data map of college students' basketball sports injuries.

**Figure 10:** Data test chart of college basketball injury model based on RBF neural network. (a) RBF neural network data map of college basketball injury data. (b) RBF neural network average data map of college students' basketball sports injuries.

**Figure 11:** Comparison diagram of two network learning models.

**Table 1:** Injuries in college basketball.

Part frequency and percentage location	Defender		Forward		Center	
	Frequency	Percentage (%)	Frequency	Percentage (%)	Frequency	Percentage (%)
Knee joint	45	21.3	58	26.4	36	23.5
Ankle joint	28	13.3	51	23.2	40	26.1
Back and spine	14	6.6	19	8.6	11	7.2
Calf	25	11.8	29	13.2	16	10.5
Hip pelvis abdominis	7	3.3	7	3.2	7	4.6
Foot	13	6.2	16	7.3	7	4.6
Pectoralis muscle	3	1.4	3	1.4	1	0.7
Wrist and forearm	16	7.6	5	2.3	5	3.2
Elbow	3	1.4	2	0.9	3	2.0
Hands and fingers	5	2.4	0	0	1	0.7
Shoulder and upper arm	13	6.2	5	2.3	1	0.7
Thighs and buttocks	14	6.6	7	3.2	4	2.7
Head and neck	9	4.3	2	0.9	6	3.9
Other	16	7.6	16	7.3	15	9.6
Total 584	211	100	220	100	153	100

**Table 2:** Sample correlation analysis.

Number of indicator groups	Indicator name	Relevance
1	Encounter pinch	0.0714
2	Heavy weight	0.0994
3	Fierce confrontation	0.0434
4	Overuse of lower extremities	0.1274
5	Midair body collision	0.0154
6	Nonstop acceleration	0.0834
7	Pull-up jumper	0.0594
8	Number of caps	0.0714
9	Lose focus	0.1074
10	Fast dribble	0.0354
11	Exercising for too long	0.1184
12	Lack of rest	0.0244
13	Shoes do not fit	0.0964
14	Drinking and smoking	0.0464

**Table 3:** Cross-check result of BP neural network.

Category	True positive rate	False positive rate	Accuracy	Feedback rate	Roc area
Severely injured	0.833	0.012	0.833	0.833	0.991
Senior injury	0.76	0.149	0.745	0.76	0.869
Moderate injury	0.763	0.075	0.795	0.763	0.913
Minor injury	0.774	0.061	0.787	0.774	0.946
Healthy	0.947	0.012	0.857	0.947	0.997
Average	0.782	0.09	0.782	0.782	0.915

## Data Availability

The data underlying the results presented in the study are included within the manuscript.

## References

[1] Shimoura K., Nakayama Y., Tashiro Y. (2019). Association between the functional movement screen scores and injuries in male college basketball players[J]. *Journal of Sport Rehabilitation*.

RETRACTED

[2] Wehsener J. (2017). Bilateral navicular stress fractures[J]. *Proceedings of the International Journal of Exercise Science: Conference Proceedings*.

[3] Helma C., Cramer T., Kramer S. (2018). Data mining and machine learning techniques for the identification of mutagenicity inducing substructures and structure activity relationships of noncongeneric compounds[J]. *J Chem Inf Comput*.

[4] Li H., Zhang M. (2021). Artificial intelligence and neural network-based shooting accuracy prediction analysis in basketball. *Mobile Information Systems*.

[5] Alderden J., Pepper G. A., Wilson A. (2018). Predicting pressure injury in critical care patients: a machine-learning model. *American Journal of Critical Care*.

[6] Wang L. (2020). Simulation of sports movement training based on machine learning and brain-computer interface[J]. *Journal of Intelligent and Fuzzy Systems*.

[7] Wang P., Gao W. (2021). Image detection and basketball training performance simulation based on improved machine learning[J]. *Journal of Intelligent and Fuzzy Systems*.

[8] Thabtah F., Zhang L., Abdelhamid N. (2019). NBA game result prediction using feature analysis and machine learning. *Annals of Data Science*.

[9] Alanis A. Y., Alma Y. (2018). Electricity prices forecasting using artificial neural networks. *IEEE Latin America Transactions*.

[10] Goel T., Nehra V., Vishwakarma V. P. (2017). An adaptive non-symmetric fuzzy activation function-based extreme learning machines for face recognition. *Arabian Journal for Science and Engineering*.

[11] Yue Q., Daley A. J., Istivan T. S., Suzanne M. G., Margaret A. D. (2017). Antibiotic susceptibility of coagulase-negative staphylococci isolated from very low birth weight babies: comprehensive comparisons of bacteria at different stages of biofilm formation[J]. *Annals of Clinical Microbiology and Antimicrobials*.

[12] Yang H., Li Z., Wang Z. (2020). Prediction of atherosclerosis diseases using biosensor-assisted deep learning artificial neuron model. *Neural Computing & Applications*.

[13] Ghahremani S., Ghanbari M. (2017). Error resilient video transmission in ad hoc networks using layered and multiple description coding[J]. *Multimedia Tools and Applications*.

[14] Schöneich S., Hedwig B. (2019). Feedforward discharges couple the singing central pattern generator and ventilation central pattern generator in the cricket abdominal central nervous system. *Journal of Comparative Physiology*.

[15] Paul S. P., Aggarwal D. S. (2021). A cognitive research tendency in data management of sensor network. *International Journal of Wireless and Ad Hoc Communication*.

RETRACTED

[16] Chen G., Lu Y., Li B. (2019). Mp-rdma: enabling rdma with multi-path transport in datacenters. *IEEE/ACM Transactions on Networking*.

[17] Wang G., Zhou J. (2021). Dynamic robot path planning system using neural network. *Journal of Intelligent and Fuzzy Systems*.

[18] Zhang D., Li W., Wu X. (2019). Application of simulated annealing genetic algorithm optimized back propagation(BP) neural network in fault diagnosis[J]. *International Journal of Modeling Simulation & Scientific Computing*.

